The article "Advances in the Study of Inhaled Formulations for the Treatment of Pulmonary Arterial Hypertension" was retracted in 2023. Reasons: signs of a paper mill; compromised peer review; unreliable results or conclusions.

# Advances in the Study of Inhaled Formulations for the Treatment of Pulmonary Arterial Hypertension

**DOI:** 10.1155/2022/6495645

**Published:** 2022-06-02

**Authors:** Fei Han, Yongqi Chen, Shijie Li, Yankun Yang, Zhonghu Bai

**Affiliations:** ^1^The Key Laboratory of Industrial Biotechnology, Ministry of Education, Jiangnan University, Wuxi 214122, China; ^2^National Engineering Research Center for Cereal Fermentation and Food Biomanufacturing, Jiangnan University, Wuxi 214122, China; ^3^Jiangsu Provincial Engineering Research Center for Bioactive Product Processing, Jiangnan University, Wuxi 214122, China; ^4^Zhuhai Resproly Pharmaceutical Technology Co., Ltd., Zhuhai 519000, Guangzhou, China

## Abstract

Pulmonary arterial hypertension (PAH) is a serious disease with reduced systemic circulation and low bioavailability associated with conventional and dosed therapy, which inhaled drugs can avoid. A mean pulmonary artery pressure (mPAP) of ≥25 mmHg (1 mmHg = 0.133 kPa) at rest or ≥30 mmHg during exercise and a pulmonary capillary pressure or left atrial pressure (PLA) of ≤15 mmHg can be diagnosed with PAH. Pulmonary hypertension is classified into primary PAH and secondary PAH according to the presence or absence of principles or risk factors. The main symptoms of pulmonary hypertension include dyspnoea, syncope, weakness, chest pain, and the presence of varying degrees of peripheral oedema. It is a highly pathogenic and life-threatening disease and can lead to delays in treatment if not diagnosed in time. In the past few years, the studies related to this progressed slowly, which brought great harm to patients with PAH. Reports showed that patients diagnosed with PAH should receive routine preventative care, such as pneumococcal and influenza vaccinations. Inhalation therapy is mainly used for the treatment of respiratory diseases and is of great interest due to the concentration of the drug in the airways and lung tissues. Therefore, the present situation of pulmonary hypertension and the characteristics of inhalation preparation were reviewed in this paper to provide some related cue for the treatment of pulmonary hypertension. In the future, it is necessary to develop more treatment methods for pulmonary hypertension.

## 1. Introduction

Pulmonary arterial hypertension (PAH) is a condition characterized by increased pulmonary vascular resistance, which can lead to right heart failure and premature death. It is a highly pathogenic and life-threatening disease and can lead to delays in treatment if not diagnosed in time [1, 2]. In the past few years, the studies related to this progressed slowly, which brought great harm to patients with PAH.

The article "Advances in the Study of Inhaled Formulations for the Treatment of Pulmonary Arterial Hypertension" was retracted in 2023. Reasons: signs of a paper mill; compromised peer review; unreliable results or conclusions.

With the continuous progress of medical treatment, its research is remarkable, such as prostacyclin and endothelin receptor antagonists, all of which have improved the quality of life of patients and reduced the death rate of the disease [3]. Pulmonary drug delivery enables direct delivery of the drug to the lung tissue, reducing the number of drugs circulating in the body and reducing the adverse effects of the drug on the patient [4, 5]. Compared to gastrointestinal drug delivery, its modality causes fewer pulmonary metabolic reactions, reduces drug damage to the liver, improves patient compliance, and avoids drug-induced complications.

Nowadays, the treatment of PAH is not so effective, which has caused great harm to patients. The purpose of this study can be itemized into 3 points: the definition and classification of PAH, the symptoms of PAH, and the treatment methods of PAH. This study will summarize the pathogenesis of PAH and search the treatment methods. The references were collected form PubMed and the keywords were “Pulmonary arterial hypertension, treatment.” We mainly focus on the advances in the treatment of patients with pulmonary hypertension using inhaled preparations, which will bring new light for future treatment.

## 2. Definition of PAH

A mean pulmonary artery pressure (mPAP) of ≥25 mmHg (1 mmHg = 0.133 kPa) at rest or ≥30 mmHg during exercise and a pulmonary capillary pressure or left atrial pressure (PLA) of ≤15 mmHg can be used to determine PAH by cardiac catheterisation. In recent years, the World Health Organization (WHO) has defined the criteria for PAH as a pulmonary artery systolic pressure > 40 mmHg (relative to a tricuspid regurgitation rate > 3.0 m/s on Doppler ultrasound). The three factors that influence pulmonary artery pressure (PAP) are pulmonary vascular resistance (PVR), cardiac output (CO), and PLA, and the relationship between the three can be expressed in the following equation: PAP = PVR × CO + PLA [3, 6].

### 2.1. PAH Classification

Pulmonary hypertension is classified into primary PAH and secondary PAH according to the presence or absence of principles or risk factors. Primary PAH is defined as pulmonary arterial hypertension except for all causes. According to the 2nd Conference on Pulmonary Hypertension held in Evian, France, experts have proposed a clinical classification of it, the main aim of which is to classify the different causes of PAH according to the same pathology and clinical manifestations [7]. The Evian classification of PAH has gained worldwide acceptance and clinical application. In the 3rd Conference on Pulmonary Hypertension, held in Venice, Italy, in 2003, the general structure and philosophy of pulmonary hypertension was maintained and modified to include idiopathic pulmonary hypertension, familial pulmonary hypertension, and pulmonary hypertension due to associated risk factors, such as connective tissue disease, congenital body-pulmonary circulation shunt disease, and HIV infection [8, 9].

The article "Advances in the Study of Inhaled Formulations for the Treatment of Pulmonary Arterial Hypertension" was retracted in 2023. Reasons: signs of a paper mill; compromised peer review; unreliable results or conclusions.

### 2.2. Signs and Symptoms of PAH

The main symptoms of pulmonary hypertension include dyspnoea, syncope, weakness, chest pain, and the presence of varying degrees of peripheral oedema. The early symptoms are not obvious, and more patients are diagnosed in the middle to late stages, but by then, the pathological and physiological changes of pulmonary hypertension have been established. [10, 11] Sarah et al. [12] showed that pulmonary hypertension (PH) is a group of pulmonary vascular diseases in which the pulmonary artery pressure exceeds a certain limit and can lead to right heart failure and even death, with a high morbidity and mortality rate, posing a serious threat to human health.

## 3. Current Status of PAH Treatment with Inhaled Formulations

The first therapy for the treatment PAH is epoprostenol, which was made available in 1995. At first, the treatment was focused on the improvements in the short term, and gradually, it has been shifted to long-term mortality-based trials. Nowadays, there are about 14 kinds of pharmacotherapeutic options which can be used for administrative routes. Reports showed that patients diagnosed with PAH should receive routine preventative care, such as pneumococcal and influenza vaccinations [13]. To improve the exercise tolerance of patients, they are encouraged to join in supervised exercise. Inhalation therapy is mainly used for the treatment of respiratory diseases and is of great interest due to the concentration of the drug in the airways and lung tissues. The high local concentration allows for a better pharmacological effect, is less costly than intravenous and oral drugs, and reduces the systemic adverse effects of the drug. Inhalation therapy has less impact on systemic adverse effects, because it is fast-acting, avoids damage to the gastrointestinal tract, and reduces metabolism of the drug in the internal organs. The following inhalation drugs are relevant to the treatment of PAH, as shown in Table 1 [14, 15]. There are several release inhalation delivery systems used nowadays, such as liposomes, biodegradable nano- and microparticles, formation of coprecipitates, and complexation with cyclodextrins [16].

### 3.1. Prostacyclin Analogues

Prostacyclin is mainly formed by vascular endothelial cells and plays an important stabilizing role in maintaining the system of the intravascular environment. Prostacyclin binds to specific membranes and simultaneously exhibits the effectiveness of effector cell receptors and, through the association of G proteins and adenylyl cyclase, is able to obtain enhanced intracellular effects of cyclic adenosine monophosphate, which effectively activates protein kinases, reduces cellular concentrations, and produces a number of biological effects, specifically shown to inhibit platelet coagulation, modulate increased inflammation, and strongly relax vascular smooth muscle [17, 18].

The article "Advances in the Study of Inhaled Formulations for the Treatment of Pulmonary Arterial Hypertension" was retracted in 2023. Reasons: signs of a paper mill; compromised peer review; unreliable results or conclusions.

Iloprost is a synthetic and relatively stable cyclin analogue with a relatively short duration of action, administered by inhalation 6-9 times a day. It has been demonstrated that the use of 100 *μ*g of iloprost in 6-9 inhalations per day for varying lengths of time, up to 1 year, in patients with different grades of PAH has been found to provide short- or long-term benefits [19]. Currently, the United States, Australia, and some other European countries have approved inhaled iloprost for direct use in the treatment of WHO cardiac class III or IV PAH, and in China, it was approved for the treatment of moderate PAH in 2006.

Treprostinil remains relatively stable at room temperature and has a long half-life, so it is usually used for subcutaneous and intravenous injections. Pain at the injection site is a common adverse effect, and inhalation studies of this drug are increasing in order to avoid a range of adverse effects. Some studies have indicated [20] that some scholars have used it in an efficacy review with iloprost and that the efficacy of the two is comparable, with iloprost reaching its peak after 8 min and travoprost reaching its peak after 18 min, but its duration of action is up to 60 min longer than that of iloprost, and it is noted that a single dose of travoprost still has a better safety profile.

### 3.2. Nitric Oxide (NO)

NO is a mixture of gases that is more soluble in water, has a short half-life, and has a variety of biological activities that are better able to inhibit platelet aggregation, smooth muscle cell proliferation, etc. NO production by vascular endothelial cells is catalyzed by NOS and further produced. [21] NO in the lungs also plays an important role in maintaining the pulmonary circulation by activating guanylate cyclase in the smooth muscle cells of the pulmonary vasculature, causing it to undergo a series of transformations that activate protein kinases, which in turn cause the physiological effect of vasodilation. It is generally accepted that in acute hypoxia, NO production by cells in the pulmonary vasculature rises sharply to compensate for increased pulmonary vascular tone and pressure, while in patients with chronic PAH, its reduced levels directly lead to pulmonary vasoconstriction and cell proliferation in patients, so timely supplementation of NO can improve pulmonary vasodilation, and it is also absorbed by better ventilated alveoli without entering nonventilated alveoli, thus improving the effect of ventilation [22, 23].

The article "Advances in the Study of Inhaled Formulations for the Treatment of Pulmonary Arterial Hypertension" was retracted in 2023. Reasons: signs of a paper mill; compromised peer review; unreliable results or conclusions.

NO inhalation is gradually being used in the treatment of PAH. mPAP decreased significantly after 40 ppm NO inhalation. Related studies have shown that NO inhalation is significantly effective for PAH caused by different factors. Some scholars believe that the inhalation dose of NO should not be too high and that the inhalation dose is not proportional to the efficacy. 100 ppm inhalation in the short term is a safe range, while large doses may produce a series of adverse events [24]. Some studies have shown [25] that rebound occurs after cessation of high doses of inhaled NO therapy, so it is important to follow a slow reduction in the dosage of NO when using it for treatment, and the development of methemoglobin and pulmonary oedema may occur when using it for treatment.

### 3.3. Soluble Guanylate Cyclase (sGC) Agonist

SGC is a key signaling enzyme in the NO-sGC-cGMP signaling pathway, which can be activated by the endogenous dilator NO to catalyze the formation of cGMP, which can act as a second messenger to regulate the related effectors downstream of the transduction pathway, mainly protein kinases, PDEs, etc., and thus regulate the corresponding physiological processes [26]. The sGC agonist enhances the sensitivity of sGC to NO and activates it in the absence of NO. Some scholars have applied it to experimental animals in inhalation tests to observe their blood pressure and found immediate pulmonary vasodilatation and high cGMP release after absorption. If the above drug is administered first and then NO is given, it can greatly increase the degree of vasodilation of NO, but further validation is needed. sGC stimulators are commonly used in the treatment of pulmonary arterial hypertension and chronic thromboembolic pulmonary hypertension [27].

### 3.4. PDE Inhibitors

Cyclic nucleotides are intracellular second messengers that play an important role in signal transduction, and PDEs mainly regulate their hydrolysis in the cell. If PDEs are inhibited, they can still exert the biological effects of cAMP and cGMP. PDEs include different species subtypes with different affinities and specificities for different substrates. It has been shown [28] that the use of PDE inhibitors in addition to inhaled prostacyclin prolongs the duration of action of prostacyclin, improves haemodynamics, and does not affect systemic arterial blood pressure or gas exchange, but the long-term efficacy of PAH treatment with PDE inhibitors alone has not been demonstrated.

The article "Advances in the Study of Inhaled Formulations for the Treatment of Pulmonary Arterial Hypertension" was retracted in 2023. Reasons: signs of a paper mill; compromised peer review; unreliable results or conclusions.

### 3.5. Rho Kinase Inhibitors

Rho kinase is a member of the serine protein kinase family and belongs to the Rho downstream target effector molecule, which mainly includes two structures, ROCK1 and ROCK2. ROCK2 is mainly found in the brain and skeletal muscle, and both are expressed in the vascular smooth muscle. ROCKs receive Rho transactivation signals, mostly at amino acid sites, and mediate a series of phosphorylation reactions of their downstream effectors, which play an important role in cell proliferation, migration, and apoptosis [29].

### 3.6. Vasoactive Intestinal Peptide (VIP)

It has been found [30] that vasoactive intestinal peptides were first isolated from the pig small intestine and are part of the pancreatin-glucagon family. It is distributed in the central nervous system and the gastrointestinal tract, but later, it was found to be widely distributed in all tissues of the body and has more biological activity, with the ability to diastole smooth muscle cells and antiproliferative effects. One study using 200 *μ*g of VIP, given 4 times to patients with IPAH, showed a mean reduction in mPAP of 13 mmHg after 3 months of continuous treatment and an improvement in clinical symptoms including haemodynamics. Siddappa and Vege [30] have shown that even non-IPAH patients can benefit from the administration of VIP drugs. However, the existing VIP inhalation substances have a short half-life and are not long-lasting, and further research in the field of formulation needs to be strengthened.

### 3.7. Adrenomedullin (ADM)

ADM is an active peptide that is mainly found in blood plasma and in various tissues and organs and is also expressed in lung tissue. It has been shown [31] that ADM can inhibit smooth muscle proliferation and migration. It was found to be increased in patients with IPAH and PH and was positively correlated with the severity of PH. With the continuous in-depth study of ADM, it is believed that it rises with the increase of pulmonary artery pressure, is a defensive response, can regulate the imbalance between constricting and diastolic substances, can maintain the stability of the pulmonary circulation, and also can stop the migration and proliferation of cells and slow down the development of PH. Some scholars have found that the use of ADM for intravenous administration to patients with PH can rapidly reduce pulmonary artery pressure in patients, but its poor vascular selectivity leads to hypotension while reducing pulmonary artery pressure [32]. Therefore, a late test using ADM inhalation was conducted in rats after single and repeated inhalation of ADM to observe its short-term and long-term therapeutic effects. The results showed that after a single inhalation, mPAP decreased significantly and cardiac output was improved, with no significant adverse effects on the body circulation. After 3 weeks of inhalation, mPAP and pulmonary vascular resistance decreased significantly. The pathological results indicated that ADM was effective in inhibiting smooth muscle thickening in rats and improved survival rate.

The article "Advances in the Study of Inhaled Formulations for the Treatment of Pulmonary Arterial Hypertension" was retracted in 2023. Reasons: signs of a paper mill; compromised peer review; unreliable results or conclusions.

## 4. Summary

In recent years, with the continuous research on the pathogenesis of PAH, more drugs have been gradually applied in clinical treatment, but it is undeniable that more drugs are accompanied by the occurrence of systemic adverse effects and short half-life defects in the treatment of PAH. Patients with PAH or suspected PAH should be referred to an expert center. The treatment of PAH should first conclude the management of comorbidities, such as sleep apnea and COPD. Moreover, supportive therapies such as diuretics, oxygen, and management of HF are needed if indicated. [3]

With the increasing understanding of disease mechanisms and treatment, effective targets for the treatment of PAH have been identified, including prostacyclin analogues, PDE inhibitors, NO, and Rho kinase inhibitors. The use of Rho kinase inhibitors could alleviate pulmonary vasculature injury induced by hypoxia-induced pulmonary hypertension by inflammatory response. The delivery of PAH therapeutic drugs via pulmonary dosing has become an effective alternative to injectable therapy. In addition, the application of novel technologies such as polymeric micro- and nano-drug delivery systems and liposomes to inhalation formulations, combining the two perfectly, is what will enable the development of safe and effective inhalation drugs for the treatment of PAH.

This study summarized the whole treatment methods of the PAH, which provides an idea for treatments. However, there are also limits to this study. First, there is no relative explanation for the occurrence mechanism underlying this. Also, this study lacks a comprehensive conclusion of the future direction. There are also some questions that need to be solved. Are there combined medical treatments for PAH which will increase the treatment rate for patients? And when can we give more attention to patients with PAH and improve their life, avoiding accidents?

In conclusion, this study presented the situation of pulmonary hypertension and the characteristics of inhalation preparation, so as to provide some related cue for the treatment of pulmonary hypertension. In the future, it is necessary to develop more treatment methods for pulmonary hypertension.

The article "Advances in the Study of Inhaled Formulations for the Treatment of Pulmonary Arterial Hypertension" was retracted in 2023. Reasons: signs of a paper mill; compromised peer review; unreliable results or conclusions.

## Figures and Tables

**Table 1:** The inhalation drugs and their function to treat PAH.

Inhalation drugs	Function
Prostacyclin analogues	Stabilize role in maintaining the system of the intravascular environment
Nitric oxide	Inhibit platelet aggregation, smooth muscle cell proliferation
Soluble guanylate cyclase (sGC) agonist	Catalyze the formation of cGMP
PDE inhibitors	Regulate their hydrolysis in the cell
Rho kinase inhibitors	Mediate a series of phosphorylation reactions of their downstream effectors
Vasoactive intestinal peptide	Diastole smooth muscle cells and antiproliferative effects
Adrenomedullin	Inhibit smooth muscle proliferation and migration

## Data Availability

The data used to support this study are available from the corresponding authors upon request.
